This article has been retracted.

# Polymethyl Methacrylate-Based Smart Microfluidic Point-of-Care Testing of Prothrombin Time and International Normalized Ratio through Optical Detection

**DOI:** 10.1155/2022/5975228

**Published:** 2022-02-18

**Authors:** Enas W. Abdulhay, Ruba E. Khnouf, Yahia M. Karain, Taqwa K. Al Omari, Nourshan M. Ebeid, Tamara H. Al Muhtaseb, N. Arunkumar, M. Thilagaraj, Gustavo Ramirez-Gonzalez

**Affiliations:** ^1^Biomedical Engineering Department, Jordan University of Science and Technology, Irbid 22110, Jordan; ^2^Department of Biomedical Engineering, Rathinam Technical Campus, Coimbatore, India; ^3^Department of Electronics and Instrumentation Engineering, Karpagam College of Engineering, Coimbatore, India; ^4^Departamento de Telematica, Universidad del Cauca, Colombia

## Abstract

The mechanical heart valve is a crucial solution for many patients. However, it cannot function on the state of blood as human tissue valves. Thus, people with mechanical valves are put under anticoagulant therapy. A good measurement of the state of blood and how long it takes blood to form clots is the prothrombin time (PT); moreover, it is an indicator of how well the anticoagulant therapy is, and of whether the response of the patient to the drug is as needed. For a more specific standardized measurement of coagulation time, an international normalized ratio (INR) is established. Clinical testing of INR and PT is relatively easy. However, it requires the patient to visit the clinic for evaluation purposes. Many techniques are therefore being developed to provide PT and INR self-testing devices. Unfortunately, those solutions are either inaccurate, complex, or expensive. The present work approaches the design of an anticoagulation self-monitoring device that is easy to use, accurate, and relatively inexpensive. Hence, a two-channel polymethyl methacrylate-based microfluidic point-of-care (POC) smart device has been developed. The Arduino based lab-on-a-chip device applies optical properties to a small amount of blood. The achieved accuracy is 96.7%.

## 1. Introduction

Blood exists in the human body in the form of liquid. The process by which this liquid turns into a gel results in a clot and is called coagulation or clotting. The formation of a clot may result in the repair of a damaged vessel through endothelial cells, platelets, fibrin, and plasma factors among which are the prothrombin and thrombin. Forming a clot depends also on vitamin K which activates different factors and proteins. On the other hand, hemorrhage and thrombosis are diseases resulting from disorders of coagulation and leading to myocardial infarction or pulmonary embolism [1–4]. Anticoagulants (e.g., vitamin K antagonists, warfarin or heparin) are used to treat and prevent blood clots.

The coagulation is initiated when damage occurs to the endothelium lining, leading to changes in platelets. The platelet's role is forming a plug at the site of injury (primary hemostasis). On the other hand, the secondary hemostasis occurs, when different clotting factors form fibrin strands to support and sustain the platelet plug [3]. In the secondary plug formation, there are two pathways, the extrinsic and the intrinsic; the former is blocked by warfarin, and the latter is blocked by heparin. Forming a clot depends widely on vitamin K. In the extrinsic pathway, vitamin K activates a factor, which turns into another factor, with the help of a different factor. One of those factors is prothrombin. If vitamin K is activated, prothrombin turns into thrombin and helps make fibrin. Warfarin is the blockage for this pathway; it stops the activation of vitamin K, as well as the formation of fibrin. On the other hand, heparin is often used acutely in the prevention of thrombosis [5].

The mechanical heart valve is a crucial solution for many patients. However, it has disadvantages like thromboembolism as well as harms due to anticoagulation aspects [5, 6]. Essential measurements of coagulation time—in patients undergoing anticoagulation therapy—are the prothrombin time (PT) and the international normalized ratio (INR) [5]. Clinical testing of PT and INR is relatively easy. However, it requires the patient to visit the clinic for evaluation purposes. Many techniques are therefore being developed to provide self-testing INR devices based on optical, ultrasonic, viscometric, and electrical transduction principles, as well as on capturing the variation in the mechanical and electrical features. Unfortunately, those solutions are either inaccurate, complex, or expensive. For example, in [7], the viscoelastic modulus of clotting blood was quantified from the temporal intensity fluctuations of speckle patterns to derive information about the blood coagulation status. However, the clotting times spanned several minutes in contrast to seconds measured by laboratory methods. In [8], blood samples were analyzed by a point-of-care prothrombin time (PT)/international normalized ratio (INR) cartridge-based i-STAT portable blood gas analyzer. Nevertheless, the feasibility of the test takes a number of strict complex requirements into account. In [9], a fully printed prothrombin time impedimetric coagulometer was used for point-of-care testing. Yet, there was a failure to achieve complete coagulation. In [10], the blood coagulation testing was conducted through a smartphone platform using the quartz crystal microbalance dissipation method. However, the cost was relatively high. In [11], real-time electrical impedimetric monitoring of the blood coagulation process was performed under temperature and hematocrit variations in a microfluidic chip. Nevertheless, the method imposes conditions about ranges of temperature and hematocrit.

Thus, the present work approaches the design of a self-monitoring polymethyl methacrylate-based microfluidic smart lab-on-a-chip that is easy to use, accurate, and relatively inexpensive. Hence, a two-channel point-of-care (POC) device [12, 13] that uses infrared light—transmitted to a small amount of blood and analyzed by Arduino—has been developed.

### 1.1. Prothrombin Time and International Normalized Ratio

The prothrombin time measures the number of seconds it takes for a clot to form in a person's sample of blood. The international normalized ratio was developed to standardize the PT to allow for monitoring of therapy across different laboratories and reagents [14]. The INR is the ratio of the patient's PT value over the geometric mean of the PT (generated from normal volunteers) raised to the power of the international sensitivity index (ISI) of the reagent. The mean normal PT value is derived from the log mean normal prothrombin time of at least twenty normal donors. ISI indicates how sensitive the reagent is—to deficiencies in the Vitamin K dependent factors—compared to the World Health Organization reference standard.

## 2. Materials and Methods

### 2.1. Used Material

Polymethyl methacrylate (PMMA) is the synthetic polymer of methyl methacrylate. This thermoplastic polymer is used as a lightweight or shatter-resistant alternative to glass and commonly called acrylic glass. In many applications, PMMA is often preferred because of its (1) moderate properties, (2) easy handling/processing, (3) low cost [15], (4) high mechanical strength, (5) high Young's modulus, (6) high scratch resistance, (7) low water absorbing capacity, which gives it a good dimensional stability, (8) good thermal stability (it can withstand temperatures up to 100°C), and (9) good optical properties. Colored PMMA varieties allow specific IR wavelengths to pass while blocking visible light.

Acrylics are unaffected by aqueous solutions of most laboratory chemicals which means that they are chemically stable with thromboplastin and also with blood. Acrylics are easily drilled, engraved, and finished with sharp car-bide-tipped tools [16].

### 2.2. Chip Dimensions

The design should ensure the blood does not return through the reagent channel. Also, the detection area should ensure good mixing between the blood and reagent. The proposed design has therefore two inputs, two channels with 60-degree angle joining together at the mixing area with 500 nm width. The blood enters the area in a turbulent flow to allow mixing. This area leads to the detection area where the components are mixed and the coagulation happens. The design is illustrated in Figure 1.

### 2.3. Chip Fabrication

In the fabrication process, the main used devices are as follows: (1) the computer numerical control (CNC) milling machine, as a milling cutter to remove material from the surface; (2) ultrasonic bath to use ultrasound in the range 20–400 kHz with suitable cleaner solvent; (3) a spin coater to deposit uniform acetylacetone on flat chips (in general, the relation between thickness of a spin coated film and the spin speed (angular velocity) squared root is inversely proportional); and (4) a hydraulic press to use a hydraulic cylinder in order to generate a compressive force.

First, the top view of the chip is drawn using AutoCAD with the desired dimensions. The AutoCAD file is then inserted into the CNC milling machine as an input. The computer converts the drawing into G-code, a language that is understood by the machine. Second, the depth is specified so that the machine can start drilling. According to the desired dimensions, a suitable drilling bit is selected and placed in its right position. Third, the drilled chip then needs to be cleaned, and thus, it is immersed completely in water in a beaker and placed for 10 minutes in the ultrasonic bath (sonicator). Fourth, for covering, a thin PMMA slide with suitable holes—for the inputs—and identical area—as the chip—is used. Fifth, acetylacetone is distributed on the cover. The cover is then placed in a spin coater for 3 seconds at a speed 2000 rpm, which helps spread the acetylacetone on the cover evenly. Sixth, the cover is placed carefully over the chip; a proper pressure is applied for 4 minutes on the covered chip using a hydraulic press device. Finally, the covered chip is left in the oven at 40°C for 24 hours before it is ready to be used. The different steps of manufacturing are presented in Figure 2.

### 2.4. Heating Requirement

Temperature factor can influence the rate of reaction as well as the concentration variation. Preanalytical variables can therefore affect the coagulation test and factor analysis results [17–19]. To minimize variability in test results due to temperature, the chip should be kept at 37°C in a heating block, but not for too long. A close monitoring via a microprocessor is therefore necessary.

### 2.5. Heating Circuit Design

N-channel IRF540 MOSFET is used to directly heat and control the temperature. The main components include the following: (1) TL431 shunt regulator (for adjustable voltage and current referencing) used to provide VREF 4.2 V. It has specified thermal stability; (2) the LM35 temperature sensor with a linear relation between output voltage and temperature; (3) TL072 as a general-purpose JFET-input operational amplifier (for comparison); (4) IRF 540 as a power MOSFET (as heat sink); (5) BC547 as an NPN bipolar junction transistor to amplify current (epitaxial silicon transistor); (6) 1N4148 diodes as small signal fast switching diodes (silicon epitaxial planar diode); and (7) a thermal ceramic resistor as a power resistor (for heating) [20].

### 2.6. Heating Circuit Mechanism and Validation

The circuit uses the transistor as a heater. It is therefore a simple on/off-type control circuit. LM35 is the temperature sensor with the measured temperature as the output. TL072 compares the voltage that VR1 sets with the output of the LM35 to turn on Q2 (the transistor) accordingly, with the positive feedback through R9 providing a small amount of hysteresis. The set temperature value is translated into voltage by 10 mV/1°C and can be measured through the noninverting terminal of the TL072. The actual temperature is also translated into voltage by the same ration and can be measured through the inverting terminal of the TL072. The LED lights up when Q2 is on. The temperature sensor LM35 and the transistor IRF540 are thermally mounted on the sample holder. Setting bias control VR3 for a Q2 current of 270 mA is sufficient to hold the cuvette at 45°C. Since the temperature sensor is positioned directly to the chip, it provides a continuous feedback to the circuit, so that any change in temperature is detected and temperature of the chip is compromised [18, 20]. Changing the voltage divider comprising R1, R2, and VR1 can modify the desired temperature range. The reference voltage is driven from a TL431 shunt regulator. The software Proteus 8 has been used herein to validate the shunt output as well as the measured ambient and desired temperatures.

### 2.7. Optical System

The optical system is based on using infrared (IR) radiation to detect fibrin clot formation and compute the INR value through the prothrombin time. A stable source (5 mm LED) with near infrared radiation has been used (940 nm) altogether with a sensitive IR receiver (5 mm photodiode). The transmitter and the receiver are brought accurately opposite to each other letting the IR radiation pass through the sample (30 *μ*L) [21]. The optical changes arise as a result of blocking IR radiation when blood clots are formed. It is worthy to note that the reflection approach has also been attempted and compared—in our work—to the transmission approach. However, the transmission technique has been adopted as (1) it gave a better correlation value with laboratory outcomes, (2) results were more stable, and (3) it needed less amount of blood sample.

### 2.8. Microprocessor

The correctly aligned manufactured chip, optical system, and heating circuit are placed in an insulated housing with dark surfaces. The optical circuit is linked to Arduino, which powers the transmitter and receiver, reads the output of the circuit, displays readings in digital form, and determines the prothrombin time and INR value according to preprogrammed algorithms.

### 2.9. Programming of Consistency Algorithm

The output of the detector ranged from low (0 output) to high (1023 output), where low values appeared when all the light from the source got transferred to the detector and high values appeared when none of the light was sensed by the detector. The adopted Arduino programmed method of PT and INR calculation is the consistency algorithm, based on the concept that the IR receiver outcome for each sample reaches a certain value at its PT and remains constant at that value for a period of time. Hence, the measured values are saved into an array. Then, PT is considered the time from the start of the reaction until the constant value first appears. INR is calculated through the formula described in the previous sections. Moreover, the program helps display the instruction messages, the calculated values, and the brief evaluation of INR—based on a typical range (e.g., [2.5-3.5])—via a monitoring screen. The program also helps in saving the results for three months in order to keep a history for the patient.

The main structures—added to the chip—are shown in Figure 3, and the overall system block diagram is illustrated in Figure 4.

## 3. Results and Discussion

The perfect running time is found to be 42 seconds; it gives a range of INR between 1.8 and 3.8 which covers both the regions of INR for patients with a mechanical mitral valve (2.5-3.5), and for patients with mechanical aortic valves (2-3). The running times in the range 35-45 seconds were tested, and the best running time (42 s) was selected based on the least drifting and the best stability of values—compared to those measured in hospital approved laboratory—in the targeted INR ranges.

Figures 5 and 6 illustrate the correlation between INR values measured by the PMMA-based POC device and those measured in a hospital laboratory, for the same twenty blood samples. The results indicate a high coefficient of determination (0.967). The main sources of deviations or errors are hematocrit, fibrinogen, and anticoagulants.

The developed PMMA-based device offers advantages compared to laboratory testing instruments: (1) managed by the patient without the availability of the professional; (2) applied to the whole blood without the need of plasma extraction; (3) managed in home or bedside; (4) gives immediate results; (5) noticeably lower cost; and (6) noticeably lower amount of blood, given that some laboratory kits necessitate up to 100 *μ*L. Also, it offers advantages compared to available POC devices [22]: (1) noticeably lower cost (10$ per test), given that some POCT cost up to 150$ per test; (2) lower amount of blood (30 *μ*L), given that some POCT necessitate up to 75 *μ*L, and (3) exploits a principle (optical) simpler than mechanical, electromagnetic, or electrochemical detection methods. Moreover, the implemented device is stable, accurate, and sensitive, with high repeatability.

The implemented point-of-care testing aids in medical diagnosis at the time and place of patient care. Hence, the testing is not wholly confined to the medical laboratory with hours or days of waiting during which time care must continue without the desired information. The developed INR testing requires only a small sample of blood by pricking the fingertip; the blood drop is then placed on a test strip and inserted into the fabricated device which analyzes the blood and displays the INR result. This can therefore help in capacity management of the hospital facilities and clinical operations as well as in providing more frequent INR testing or eventually INR self-testing and patient self-management.

It is worthy to mention that several chip configurations were tested before selecting the optimum final choice. The first design had two inputs: one for the reagent and the other for blood. Those inputs were leading to two channels with 500 *μ*m width. The channels lead to the detection area where the reaction (coagulation) happens. This design did not satisfy the requirements because the blood kept returning back through the reagent channel. The second design had two inputs, two channels with 500 *μ*m width and a detection area where the reaction happens. That design could not ensure adequate mixing between blood and reagent. The third tested configuration (presented herein) is the optimum. Moreover, different materials were tested to develop chips through which the blood and the reagent are inserted and brought together to start the reaction. PMMA showed the optimum outcomes with a density 1.15-1.19 g/cm^3^, water absorption 0.3-2%, hardness (Rockwell M) 63-97, tensile strength (ultimate) 47-79 MPa, transmission 80-93%, and refractive index 1.49-1.498.

In the present work, the measurement of clotting time has also been studied in different temperatures to evaluate the performance of the fabricated device as well as to examine the effect on coagulation factors. The lowest PT was found at 40°C, while the highest PT was found at 45°C due to the fall in coagulation action in the plasma and to the partial inactivity of reagent. The analysis of the heating circuit through different temperatures was also conducted by the software Proteus8. The values of the resistors of the shunt regulator were chosen as 2.2 kΩ and 3.3 kΩ, respectively, according to the theoretical formula, in order to give the desired output.  Figure 7 illustrates the final circuit design.

The suggested approach proposes the consideration of infrared sensors in particular because: (1) they do not need complex conditions to work stably compared to other sensors that may suit our application, (2) IR sensors are cheaper than the photoresistors used to detect laser, (3) the targeted application does not require detection from long distances, and the IR receiver is therefore suitable, and (4) the aimed infrared application has shown good sensitivity, accuracy, and stability. Nevertheless, the coupling of transmitter and receiver should be carefully implemented. In the present work, the IR LED is powered by 5 V and is supposed to emit infrared radiation when a small current passes through it. The continuous forward current for IR LED is 100 mA, which is the maximum current value that the LED can handle. The IR LED forward voltage equals 1.4 V. According to the IR LED specifications, the minimum value for the resistor connected in series with it is 36 *Ω*. To restrict the current passing through the IR LED, an 150 Ω resistor is placed as a current limiting resistor to limit the diode drive current in order to provide a sufficient beam intensity to detect the coagulation process. On the other side, the IR photodiode changes its internal resistance when exposed to IR radiation. It is reversely biased and wired in series with a 10 kΩ resistor. The photodiode has a high sensitivity at the operating wavelength of the transmitter, which is 940 nm. The output is taken across the IR photodiode. Therefore, the level of the output voltage is determined by the ratio of the 10 k resistance to the resistance of the IR receiver (voltage division). As the IR photodiode receives more infrared radiation from the IR LED, its resistance decreases, therefore producing smaller output voltage. Practically, the proposed optical circuit is capable of detecting the received IR radiation during the coagulation process.

The introduced optical system can be easily customized to detect the coagulation process using two different approaches. The first approach determines the prothrombin time by optically detecting the decrease in IR radiation transmitted to the IR photodiode as the coagulation process starts. That is the transmission approach. In contrast, the second approach relies on the increase in the amount of reflected IR radiation, which is detected by the IR photodiode to measure the prothrombin time, therefore, called the reflection approach. Decisively, each optical approach implies a different positioning for the transmitter and the receiver. In the presented work, transmission showed more accurate results compared to reflection (Figures 5 and 6). The coefficient of determination (*R*^2^) for transmission measurements is larger which means less variance. After removing the outliers, the transmission gave an accuracy of 96%+, where the reflection method gave only 85%. In addition, transmission enabled the measurement using a smaller amount of blood (30 *μ*L), whereas in the reflection method, 50 *μ*L blood volume was needed to perform the test. Transmission also showed more stable results while in reflection, there were unwanted fluctuations during the same measurement.

The consistency algorithm gives the optimum results among a number of tested algorithms. At first, observing the output of the detector gave an idea that the blood sample changes the amount of light sensed by the detector as clotting starts, and the values tend to go towards the high values as the sample clots more. This gives rise to the idea of having a limit value close to the high value, and the PT time is measured from the moment the reaction starts until this value appears. The downside to this algorithm was that blood samples with different PT time and INR reached different limits; thus, one fixed limit was not enough to apply to all the samples. Another algorithm was tested by comparing every value given by the detector—every half a second—with the value before, and if the difference in their outputs exceeds a certain threshold, then the PT time is measured from the moment the reaction starts until this threshold occurrence. However, samples have different thresholds.

All of the elements mentioned above lead to the proposed device that satisfies the targeted requirements.

## 4. Conclusion

The proposed microfluidic design offers an accuracy of about 96% for INR and PT measurements. The measured values are in the range 1.8-3.8, which includes the INR values for the targeted patients. The presented device is cheaper and simpler than other POC devices on the market, and it necessitates less blood volume. Also, it offers the bedside testing that cannot be provided by current methods established in hospital analysis laboratories.

The presented work offers a promising accurate, simple, and low-cost POC technique that helps measure INR and PT via a microfluidic chip and through optical measurement. This is very useful for patients under anticoagulation treatments who need frequent monitoring but cannot visit the laboratory daily or wait for long days before getting the blood analysis results.

The future perspectives are the improvement of accuracy, the miniaturization of the whole system, and the validation on several ranges of PT/INR.

## Figures and Tables

**Figure 1:** Final chip design.

**Figure 2:** Fabrication process steps. (a) AutoCAD dimensions. (b) CNC milling machine. (c) Drilling process. (d) Ultrasonic bath. (e) The chip and its cover. (f) Spin coater. (g) Hydraulic press. (h) Fabricated chip.

**Figure 3:** Main structures. (a) Optical system. (b) Heating circuit. (c) Consistency program. (d) Arduino microprocessor.

**Figure 4:** Block diagram of the overall system.

**Figure 5:** Correlation between INR measured by the implemented device and in the laboratory.

**Figure 6:** Correlation between INR measured by the implemented device and in the laboratory (reflection method).

**Figure 7:** The optimum design of heating circuit (presented via Proteus8).

## Data Availability

The data is available only upon valid request.
